# Quality Evaluation Model for Smart City Social Sports Information Cloud Service

**DOI:** 10.1155/2022/4064747

**Published:** 2022-01-12

**Authors:** Lan Zhang

**Affiliations:** Department of Sports and Arts, Zhejiang Yuexiu University, Shaoxing 312000, China

## Abstract

With the continuous development of social economy, social sport is more and more valued and favored by the people as a universal and nationwide sport, but it should be noted that social sport involves a wide range of aspects, but due to its particularity, it is also constrained by economic development. In view of these needs and limitations, three technical methods of entropy method, RSR (rank-sum ratio), and TOPSIS are introduced, to sort out the development of social sports, national physical development, social sports guidance, and the number of people to be measured in various places based on the relevant technologies of smart cities in this paper, realize the application analysis of social sports in the public service level. This paper aims to provide a scientific evaluation and evaluation method for social sports information cloud services. The results of simulation experiments show that the evaluation of social sports information cloud service quality based on smart cities is effective, and the comprehensive application of methods can be implemented perfectly, and the further promotion and popularization of social sports services can be realized.

## 1. Introduction

With the continuous development of social economy, physical exercise has become the main way of sports that people are more enthusiastic about, such as running, climbing, and cycling [1, 2]. On the one hand, sports can improve the physical fitness of everyone but also can ensure the popularization of sports methods. For social sports, it is a systematic project, covering a wide range; meanwhile, with the development of the economy, its connotation and corresponding content have changed, especially relative to the subjective judgment of the people [3, 4]. Therefore, how to effectively and objectively evaluate social sports is a problem to which industry scholars attach great importance [5, 6]. Many scholars have tried to conduct evaluation research of social sports from different perspectives, such as constructing a five-dimensional index system of government responsibility, investment, service benefits, social feedback, and value of social sports services. Through iterative calculation of methods, comprehensive evaluation is performed, such as constructing an index system covering public participation satisfaction, public service input, efficiency, etc., using AHP method to evaluate social sports services, and providing corresponding decision support for government decision-making [1, 7]. In addition, some scholars conduct surveys, statistics, and analysis of different residents based on whether the audiences they serve are satisfied through questionnaires, visits, and consultations and other methods to reflect the popularity of social sports development from the perspective of the audience and whether there are many problems in the enjoyment of the audience, etc. [8, 9].

However, it is worth noting that, due to the restrictions and limitations of data sources, these studies are often conducted based on surveys, visits, questionnaires, etc. The audience's thinking time and response time are relatively concentrated or less, so the survey result may not completely represent their own true feelings [10, 11]. The development of cloud computing, Internet of Things, big data, and other technologies has promoted the continuous improvement of data collection, storage, analysis, mining, and other technologies. To a certain extent, it can solve the problem of shortage of manpower, less data sharing, unbalanced equipment, and the limited right enjoyed by audience [12, 13]. Therefore, in view of these needs and limitations, the “Internet +” technology is introduced by trial in this paper, through the use of entropy method, rank-sum ratio method, TOPSIS, and other three technical methods, combining the status quo of social sports public services, in order to construct the corresponding social sports service evaluation index, to promote the transformation of social sports from traditional artificialization *l* to intellectualization, explore and solve the problems encountered by the people in social sports, and aim to improve the quality and effect of the public services of social sports for the people.

## 2. Research Objects and Methods

### 2.1. Research Object

The effectiveness of the method under the smart city technology can be verified through selecting certain 11 areas of the experimental area as the research object of the social sports public service level.

### 2.2. Research Method

By selecting the corresponding latest survey data, the development level of social sports, the number of people to be tested for national physique, the number of sports activities in the year, social sports groups, and other indicators are analyzed, compared, and calculated through selection and integration of corresponding current survey data, integration of Internet mobile phone signaling data, statistical yearbook data, and other data for summary, and the specific statistical results are shown in Figure 1.

For the analysis of social sports indicators, quantitative and qualitative analysis can be carried out in the following ways, including literature method, consultation and interview method, field investigation, and practical analysis method [12, 13]. Among them, the literature method is for summarizing, sorting, and analyzing, to provide a research basis and ideas for quantitative analysis of corresponding indicators by use of existing academic papers, public news reports, and other materials, while the interview method is to obtain the corresponding attitude and understanding of social sports services through the direct communication with audience or corresponding field experts about some questions [14, 15]. On-site inspections are to conduct on-site investigations of residents through visits and reading materials to obtain the most direct evaluation based on the distribution of equipment related to social sports [16, 17]. The logical approach is to conduct analysis and inverting according to the collected relevant data and finally get the corresponding index evaluation analysis.

Based on clarifying the relevant coverage of the index, the corresponding evaluation and analysis are carried out continuously.

#### 2.2.1. Entropy Method

The entropy method is an objective and weight-based method, which is used to confirm and calculate the weight of the corresponding index. For diversified metrics, entropy is a specific method that can determine the weight. Because of these abovementioned characteristics, it can be used to clarify the weight determination of social sports and determine the weight evaluation value of social sports public services through the corresponding data sequence.

To conduct an effective social sports cloud service quality evaluation, the specific steps are mainly as follows:

(1) Orienting at the test area: a diversified evaluation index of social sports is constructed, and a matrix is used to make judgments, among which, *R*=(*X*_*ij*_)_*nm*_, (*i*=1,2,…, *n*; *j*=1,2,…, *m*).
(2) Normalize the judgment matrix *R* to obtain the normalized judgment matrix *R*′=(*Y*_*ij*_)_*nm*_.
The larger the value of the evaluation index, the better in this research. Therefore, the calculation formula is shown as follows:
  (1) $$\begin{array}{c} Y_{ij}=\frac{x_{ij}-x_{\min}}{x_{\max}-x_{\min}}. \end{array}$$
According to formula (1), the normalized matrix is calculated as
  (2) $$\begin{array}{c} Y_{ij}=\left[\begin{array}{ccccccccc} 0.3011 & 0.5861 & 1.0000 & 0.0000 & 0.0203 & 0.3031 & 1.0000 & 1.0000 & 0.3832\\ 0.5774 & 0.3483 & 0.2853 & 0.1792 & 0.1874 & 0.4492 & 0.0411 & 0.0432 & 0.5661\\ 0.3962 & 1.0000 & 0.1982 & 0.0255 & 0.0911 & 0.0000 & 0.0072 & 0.0022 & 0.4152\\ 0.000 & 0.3722 & 0.1113 & 0.7694 & 1.0000 & 0.8104 & 0.0593 & 0.1242 & 0.8862\\ 0.5771 & 0.2412 & 0.0681 & 0.1532 & 0.0451 & 0.9321 & 0.1360 & 0.0483 & 1.0004\\ 1.000 & 0.7011 & 0.8243 & 0.6151 & 0.0242 & 0.554 & 0.3392 & 0.3041 & 0.7865\\ 0.9311 & 0.1511 & 0.0251 & 0.0253 & 0.0372 & 0.5882 & 0.0000 & 0.0000 & 0.4526\\ 0.8445 & 0.1159 & 0.1586 & 1.0000 & 0.0000 & 0.3956 & 0.1053 & 0.0171 & 0.7422\\ 0.3792 & 0.1443 & 0.1051 & 0.3331 & 0.0021 & 0.2875 & 0.0064 & 0.0021 & 0.4713\\ 0.9911 & 0.3235 & 0.3972 & 0.9482 & 0.4011 & 1.0000 & 0.0172 & 0.0012 & 0.5413\\ 0.3101 & 0.0000 & 0.0000 & 0.1021 & 0.0222 & 0.5314 & 0.0080 & 0.0063 & 0.0000 \end{array}\right]. \end{array}$$
(3) The calculation formula for calculating the entropy of the *j*th evaluation index is shown as follows:
  (3) $$\begin{array}{c} H_{j}=\frac{1}{\ln\;n}\left(\sum_{i=1}^{n}f_{ij}\ln\;f_{ij}\right). \end{array}$$
Among them, it can be calculated by
  (4) $$\begin{array}{c} f_{ij}=\frac{1+Y_{ij}}{\sum_{i=1}^{n}\left(1+Y_{ij}\right)}. \end{array}$$
(4) Carry out the sparse calculation of entropy weight on the basis of formula (4). The specific calculation formula is shown as follows:
  (5) $$\begin{array}{c} w_{j}=\frac{1-H_{j}}{m-\sum_{j=1}^{m}H_{j}}, \end{array}$$
(∑_*j*=1_^*m*^*w*_*j*_=1; 0 ≤ *w*_*j*_ ≤ 1). The calculated entropy weight coefficient is the weight.

Based on the above calculation steps, the determined weights of the evaluation indicators are shown in Figure 2.

#### 2.2.2. TOPSIS Method

The TOPSIS method is a diversified decision-making method, which uses the distance between the positive and negative TOPSIS and the object to be measured for quantitative evaluation and ranks them correspondingly in terms of superiority and inferiority, which is extremely effective in multiobjective decision-making [18, 19].

The TOPSIS method is a multiattribute decision-making method. Its basic idea is to sort the advantages and disadvantages by calculating the distance between the evaluation object and the TOPSIS (*X*^+^) and negative TOPSIS (*X*^−^). According to this method, only each utility function is required to have the monotone increasing (or descending) characteristics, which is a commonly used effective method in multiobjective decision analysis.

#### 2.2.3. RSR Method

The rank-sum ratio method is to obtain a dimensionless statistic RSR through rank conversion in a matrix of *N* rows and *M* columns (*M* evaluation indicators) and rank the advantages and disadvantages of evaluation objects according to the RSR value.

First, a data analysis matrix for different evaluation indicators of social sports oriented at the experimental area is constructed. Because different evaluation indicators have different meanings and dimensions, the indicators are required to be normalized to achieve unified contrast and comparison. The specific normalization processing is shown in the following formula:

(6) $$\begin{array}{c} Z_{ij}=\frac{X_{ij}}{\sqrt{\sum_{i=1}^{16}{\left(X_{ij}\right)}^{2}}}. \end{array}$$

In the formula, the value range of *i* is [1, 11], and the value range of *j* is [1, 9]. According to the above formula and method, the matrix of the normalized evaluation index of social sports public service level is solved, and the specific expression is expressed by *Z*:

(7) $$\begin{array}{c} z=\left[\begin{array}{ccccccccc} 0.2901 & 0.3844 & 0.7042 & 0.0253 & 0.0242 & 0.1842 & 0.9121 & 0.9453 & 0.1921\\ 0.3012 & 0.2314 & 0.2013 & 0.1232 & 0.1752 & 0.2438 & 0.0622 & 0.0515 & 0.2752\\ 0.2941 & 0.6504 & 0.1394 & 0.0413 & 0.0912 & 0.0611 & 0.0321 & 0.0132 & 0.2044\\ 0.2782 & 0.2471 & 0.0795 & 0.4381 & 0.9023 & 0.3922 & 0.0853 & 0.1261 & 0.4221\\ 0.3012 & 0.1624 & 0.0482 & 0.1092 & 0.0523 & 0.4424 & 0.1542 & 0.0513 & 0.4723\\ 0.3181 & 0.4592 & 0.5815 & 0.3565 & 0.0321 & 0.2832 & 0.3352 & 0.2941 & 0.3714\\ 0.3151 & 0.1062 & 0.0182 & 0.0412 & 0.0442 & 0.3013 & 0.0362 & 0.0141 & 0.2251\\ 0.3124 & 0.0813 & 0.1121 & 0.5613 & 0.0111 & 0.2223 & 0.1231 & 0.0223 & 0.3523\\ 0.2932 & 0.1032 & 0.0743 & 0.2054 & 0.0121 & 0.1761 & 0.0341 & 0.0123 & 0.2331\\ 0.3181 & 0.2181 & 0.2806 & 0.5341 & 0.3632 & 0.4703 & 0.0452 & 0.0142 & 0.2642\\ 0.2903 & 0.0072 & 0.0002 & 0.082 & 0.0312 & 0.2752 & 0.0362 & 0.0132 & 0.0242 \end{array}\right]. \end{array}$$

## 3. Simulation Experiment

It is not only a reform of business management, but also a reform and improvement of external services *z*=[] to introduce cloud computing technology into the social sports management business. The improvement of these two aspects requires the transformation of traditional social sports and services from passive mode to active one. The corresponding social sports intelligent subject service system is designed in this paper, and the specific structure is shown in Figure 3.

According to the overall architecture shown in Figure 3, the social sports smart service system constructed in this article is mainly divided into three parts, which are distinguished as cloud providers, social sports management business personnel, and users according to different object-oriented aspects, respectively. When constructing a social sports smart public service system, full consideration should be given to the application requirements of users as the most basic and the largest number of users.

Based on the overall architecture, it is necessary to consider the hardware and software environment required for deployment. The infrastructure mainly includes hardware environments such as servers and storage, as well as operating network environments, disaster recovery backups, etc. These software and hardware environments need to be fully utilized; construct the cloud service platform accordingly with this technology. The specific process diagram is shown in Figure 4.

As shown in Figure 5, the first is the cloud layer, which is the layer that relies on cloud infrastructure. It mainly provides storage, hardware, memory, and other environments. With these infrastructures, the integrity and security of the platform can be ensured. Transfer of service providers need to be carried out in the middle of the cloud for the social sports, to coordinate the management of users and service owners and provide external services on mobile terminals or PC terminals through the network environment.

The next is the library layer of the model. This part is to realize the relationship between social sports itself and users. The schematic diagram is shown in Figure 5. Through the analysis of user needs, it ensures that the service has comprehensively changed orientating at the actual social sports and user needs. For the services provided by social sports, users have highlighted individual needs, which requires cloud computing to give full play to its advantages and provide more demanding needs. In this context, based on cloud computing technology, the cloud platform of social sports can analyze user interests, adjust service goals of social sports, and optimize service methods and content based on habits and browsing history of users.

The last is the user layer. For social sports, users are the foundation and core of the entire platform. According to users' information sharing and use, to achieve the purpose of learning and creation, their individual needs should be fully considered.

According to the data collected above, the ideal positive and negative solutions in the evaluation indicators of the social sports information cloud service quality of smart cities can be calculated.

### 3.1. The Low Actual Executive Force of Urban Community Sports Public Service Policies and Regulations

The public service quality evaluation of social sports according to the corresponding community is shown in Figure 6.

From the results, it can be seen that the proportion of residents being very satisfied is less than 10%, the proportion of being relatively satisfied is about 30%, and the sum of general and dissatisfied residents has exceeded 50%. From the collected data, it can be seen that corresponding policies are not implemented for social sports, and there are some weaknesses in publicity and popularization. Therefore, the residents are not satisfied with the quality of public services of social sports.

It can be seen from Figure 7 that most of the funding sources of social sports are government investment and support, and a small amount of funding comes from corporate donations. Therefore, most of the social sports venues still require a large amount of investment. It is precisely because of the insufficient funding that there are fewer public service facilities for social sports and the reduction of service experience.

### 3.2. The Low Implementation Speed and Efficiency of Urban Social Sports Public Services

The so-called implementation efficiency of urban community sports public services refers to whether the principal part of urban community sports public services can efficiently satisfy the public's various sports needs in the process of providing various sports services to the public.

Through investigation and research, it is found that there are obvious regional differences in the quality of social sports public services in cities, which are restricted by local social development. For example, in areas with more developed economies, the efficiency and quality of public services for social sports are relatively satisfactory and can basically meet the needs of social sports of various audiences, but the relative execution efficiency in other areas is significantly lower.

In the construction of cloud service platform guarantee capacity, virtualization technology is the core technology for cloud resource management, scheduling, and transformation into platform guarantee capacity. In platform construction, virtualization technology should be used to realize on-demand allocation and unified scheduling of cloud resources, to strengthen the fine-grained division of infrastructure resources, cloud computing resources, cloud storage resources, cloud system platform resources, and cloud software resources, and to combine services. The characteristics of the object and service content, adopting different management standards, allocation strategies, packaging methods, and usage methods, really strengthen the management and control efficiency of virtual resources; secondly, the application security, reliability, and trustworthiness and reliability of the cloud service platform should be improved. Verification, under the premise of ensuring the cloud service provider has a high degree of credibility and security, realizes the dual identity authentication and security management of the cloud service provider and the platform user; third, the compatibility of the cloud service platform system and software should be strengthened. Availability, support of sports cloud services, availability of cloud applications and databases, cloud service migration capabilities, and capacity building ensure that traditional sports can efficiently, safely, orderly, and economically migrate to the cloud computing environment according to the athletes' cloud use needs. In the construction of the IaaS service platform, the user's ease of use and manageability of IaaS resources should be emphasized to ensure that users can obtain IaaS resources through Web application services. At the same time, administrators can use the IaaS platform monitoring and management system to quickly realize the creation, deployment, allocation, scheduling, management, and monitoring of IaaS resources and ensure the load balance of the IaaS cloud service platform; secondly, the intelligence of the IaaS service platform resources should be strengthened. Dispatching and automated scheduling capabilities ensure that users can dynamically use resources in an efficient, flexible, scalable, and automatic way according to cloud application requirements and reduce usage costs by paying for usage; third, the IaaS service platform should have a larger system scale and application. Security, through the management and monitoring of resource pools, user resource allocation and scheduling, resource pool architecture optimization, and refined application operations of data transmission guarantee networks and the intensive management of IaaS cloud resources can be realized to ensure the security, efficiency, and efficiency of the IaaS platform, hostable and easy to expand. In the cloud computing environment, the data center has the characteristics of complex infrastructure structure, difficult management of cloud platforms and application systems, increased threats from the Internet, and cloud service platform resources shared by multiple users, and the cloud platform application service system is in a complex network environment middle. At the same time, cloud computing resources are logically divided and shared by multiple users in the distribution and use methods, leading to malicious users who may obtain control rights of the cloud system platform through illegal means and steal important data and user confidential information of the cloud system.

### 3.3. Failure to Give Full Play to the Role of Sports Clubs and Lack of Fitness Guidance

With the development of social economy, social sports corporation plays an important role in the important process of sports popularization and sports reform.

As shown in Figure 8, social sports groups do not fully cover the audience. Many residents do not even know about such organizations, accounting for about 30%. A small number of people participate in social sports activities. From the results in Figure 8, it is found that the audience is not very enthusiastic about participating in the corresponding social organizations.

As the core of social sports, social sports instructors play an important guidance role in public services. From the summary results in Figure 9, it can be found that, in the actual guidance process, those exceeding 6 times account for about 15%, which shows the role of social sports instructors in the actual operation process is too weak, which restricts the audience's enthusiasm for participating in sports.

### 3.4. The Low Type, Frequency, and Participation of Urban Community Sports Public Service Activities

The proportion in population of sports that young people like is relatively small. Due to the limitation of venues and equipment, the development of this type of sports is restricted. Community sports public service departments should consider increasing the construction of venues and equipment to increase the number of people participating in community sports, meet the needs of various groups of people, and continuously improve the quality of urban community sports services.

### 3.5. Calculate the Distance between Each Evaluation Index Data and *X*^+^, *X*^−^

The calculation formula for the distance *d*_*i*_^+^, *d*_*i*_^−^ between each evaluation index data and *X*^+^, *X*^−^ is shown in the following formulae:

(8) $$\begin{array}{c} d_{i}^{+}=\sqrt{\sum_{j=1}^{9}{\left(Z_{ij}^{\prime }-X_{j}^{+}\right)}^{2}}, \end{array}$$

(9) $$\begin{array}{c} d_{i}^{-}=\sqrt{\sum_{j=1}^{9}{\left(Z_{ij}^{\prime }-X_{j}^{-}\right)}^{2}}, \end{array}$$

where *i* = 1, 2, 3,…, 16 and *j* = 1, 2, 3,…, 8.

Based on this, the public service level of sports is evaluated and ranked. The specific calculation is shown in formula (10), and some results are shown in Figure 10:

(10) $$\begin{array}{c} C_{i}=\frac{d_{i}^{-}}{d_{i}^{+}+d_{i}^{-}}, \end{array}$$

where *i* = 1, 2, 3,…, 16.

Through simulation experiments, the results show that the variance consistency between the classifications of each indicator is relatively good, and the differences between the files are statistically significant, and the evaluation of social information cloud service quality under the background of smart cities is effective.

1. Build a national fitness social sports information service cloud platform that includes public and private clouds, and divide social sports cloud storage into corresponding public cloud storage and private cloud storage: public cloud is built on the Internet, and social sports management is built on a private cloud. In the government Intranet, all kinds of social sports management data are published on the Internet and Intranet through the form of services and can be integrated with various services such as government affairs and office running in the local area network and wide area network, so as to achieve the sharing of social sports management information and computing resources. The goal of the cloud platform can also provide a full range and multiangle for different users such as the State Sports General Administration, the Provincial Sports Bureau, the Municipal Sports Bureau, the Sports Guidance Center, the sports fitness site, the fitness team, the sports instructor, the seller, the sports venue, and the general public service.
2. Build a national fitness social sports big data center, and store site information, social instructor information, training methods, training information, and other structured and unstructured information on a big data platform (HDFS, HBase, etc.) to form an authoritative large-scale database covering all aspects of national fitness and social sports to provide data sources for national fitness management, resource allocation, fitness guidance, and fitness evaluation. An authoritative large database covering all aspects of national fitness and social sports serves as a data source for national fitness management, resource allocation, fitness guidance, and fitness evaluation.
3. Focus on the four core issues of fitness venues (“where to practice”), fitness people (“who will practice”), social instructors (“who to practice”), and fitness methods (“how to practice”), the design includes basic data management, information collection, data management, data query, data visualization, statistical analysis, data mining, decision support, and other major functions of the city's national fitness social sports information service system.
4. Use object-oriented programming language to develop the corresponding C/S mode background management system (C# language), B/S mode online service website (C# language), and mobile phone APP software (Java language), supporting two-dimensional code scanning is free to download and update automatically. Both the website and the mobile APP can quickly access various fitness project guidance materials (“how to practice”), and the management system is responsible for the maintenance and management of “where to practice,” “with whom to practice,” and “how to practice” related information. The actual application effect of the platform shows that the information platform has completed the foundation of 2,697 fitness sites and 21,295 social sports instructors at all levels in Dalian (84, 1731, 6,989, and 13,421 people at the national, first, second, and third levels). Information management greatly reduces the workload of managers and at the same time provides millions of intelligent information services for tens of thousands of fitness people. Users access the cloud platform through desktop systems, websites, and mobile apps (Android) and use cloud map services and cloud information services among them. In the subject of “who will practice,” the public can use interactive applications such as online quick query to solve “where to practice” (find sites/venues), “with whom to practice” (recommend social instructors based on fitness programs), and “how to practice” (push learning materials according to fitness programs). Search for fitness sites, instructors, fitness paths, etc. based on location-based services through maps, and select the best fitness activities, fitness venues, and travel methods.
5. The social sports service platform designed and constructed based on cloud computing, “Internet +,” and other technologies is essentially a loosely coupled architecture, which can be flexibly connected with existing systems and new systems in the future and ultimately can achieve “data in the cloud.” The new application service model of “sports by your side, applied in your hands” can satisfy the internal service model and external service model. “Unmanned guidance” issues practically introduce cloud computing, big data, Internet + and other thinking and technical methods into national fitness services, realize the transformation of national fitness services from artificial to intelligent, and effectively improve the public service quality of national fitness.
6. Provide a reference for building an “Internet +” smart sports information service platform with authoritative data support and persistent services, and ultimately make it a part of smart sports and smart cities.

## 4. Conclusions

With the continuous development of social economy, people are paying more and more attention to sports. As a national sport, social sports public service industry is valued. Aiming at how to evaluate social sports public services, the relevant technologies of smart cities is introduced in this paper, based on TOPSIS, rank-sum ratio, entropy method, and other methods, social sports instructors, the number of people to be tested, and other analysis index systems are constructed by trial, and they are divided by classifying, to explore the public service level of social sports, aiming to explore the evaluation of cloud service quality of social sports information in the context of smart cities. The simulation results show that the relevant technologies of smart cities are effective, can support the quality evaluation of social sports information cloud service, and can promote the further popularization of social sports.

## Figures and Tables

**Figure 1:** List of evaluation index values of social sports public service level in some regions.

**Figure 2:** Entropy weight of evaluation index for sports public service level.

**Figure 3:** The overall architecture of the cloud service platform.

**Figure 4:** Cloud service platform model.

**Figure 5:** Schematic diagram of social sports interaction (taking borrowing sports books from library as an example).

**Figure 6:** Statistics of residents' satisfaction with the quality of public services of community sports (*N* = 600).

**Figure 7:** Main sources of service funding of community sports (*N* = 12).

**Figure 8:** Statistics on the frequency of community residents participating in club activities.

**Figure 9:** Statistics of the number of times that city community fitness instructors give community guidance.

**Figure 10:** List of *C*_*i*_ values and rankings of sports public service levels in some regions.

## Data Availability

The labeled dataset used to support the findings of this study is available from the corresponding author upon request.

## References

[1] Wang X., Sheng B., Zhang C., Xiao Z., Wang H., Zhao F. (2018). An effective application of 3D cloud printing service quality evaluation in BM-MOPSO. *Concurrency & Computation Practice & Experience*.

[2] Manuel P. (2015). A trust model of cloud computing based on quality of service. *Annals of Operations Research*.

[3] Wang Y., Wen J., Wang X., Zhou W. (2017). Cloud service evaluation model based on trust and privacy-aware. *Optik-International Journal for Light and Electron Optics*.

[4] Yaghmaee M. H., Banaee F., Seno S. (2019). Performance evaluation of CoAP proxy virtualization in cloud-assisted sensornetworks. *IET Wireless Sensor Systems*.

[5] Duan Q. (2016). Cloud service performance evaluation: status, challenges, and opportunities-a survey from the system modeling perspective. *Digital Communications & Networks*.

[6] Xia Y., Zhou M., Luo X., Zhu Q., Li J., Huang Y. (2014). Stochastic modeling and quality evaluation of infrastructure-as-a-service clouds. *IEEE Transactions on Automation Science & Engineering*.

[7] Hao H., Zhang J. The evaluation system for cloud service quality based on SERVQUAL.

[8] Leung V. C. M., Shami A., Liao L. (2015). Distributed flowvisor: a distributed flowvisor platform for quality of service aware cloud network virtualisation. *Networks IET*.

[9] Labidi T., Mtibaa A., Brabra H. (2016). CSLAOnto: a comprehensive ontological SLA model in cloud computing. *Journal on Data Semantics*.

[10] Greenspan S. L., Singer A., Vujevich K. (2018). Implementing a fracture liaison service open model of care utilizing a cloud-based tool. *Osteoporosis International*.

[11] Wang Y., Xin Z., Yang D. (2017). Evaluation methodology for fast switching cloud RAN systems. *IEEE Communications Letters*.

[12] Anisetti M., Ardagna C., Damiani E., Gaudenzi F. (2017). A semi-automatic and trustworthy scheme for continuous cloud service certification. *IEEE Transactions on Services Computing*.

[13] Yang Y., Yang B., Wang S., Liu W., Jin T. (2019). An improved grey wolf optimizer algorithm for energy-aware service composition in cloud manufacturing. *International Journal of Advanced Manufacturing Technology*.

[14] Cappanera P., Paganelli F., Paradiso F. (2019). VNF placement for service chaining in a distributed cloud environment with multiple stakeholders. *Computer Communications*.

[15] Benbrahim S.-E., Quintero A., Bellaiche M. (2019). Live placement of interdependent virtual machines to optimize cloud service profits and penalties on SLAs. *IEEE Transactions on Cloud Computing*.

[16] Mubarok K., Xu X., Ye X., Zhiong R. Y., Lu Y. (2018). Manufacturing service reliability assessment in cloud manufacturing. *Procedia CIRP*.

[17] Anitha R., Mukherjee S. (2015). “MaaS”: fast retrieval of data in cloud using metadata as a service. *Journal of Intelligent Manufacturing*.

[18] Nastic S., Truong H. L., Dustdar S. (2015). SDG-Pro: a programming framework for software-defined IoT cloud gateways. *Journal of Internet Services & Applications*.

[19] Kar A. K., Rakshit A. (2015). Flexible pricing models for cloud computing based on group decision making under consensus. *Global Journal of Flexible Systems Management*.

